The article "Combined Effect of Famine Exposure and Obesity Parameters on Hypertension in the Midaged and Older Adult: A Population-Based Cross-Sectional Study" was published in 2021. Journal: Biomed Res Int.

# Combined Effect of Famine Exposure and Obesity Parameters on Hypertension in the Midaged and Older Adult: A Population-Based Cross-Sectional Study

**DOI:** 10.1155/2021/5594718

**Published:** 2021-09-23

**Authors:** Lin Zhang, Liu Yang, Congzhi Wang, Ting Yuan, Dongmei Zhang, Huanhuan Wei, Jing Li, Yunxiao Lei, Lu Sun, Xiaoping Li, Ying Hua, Hengying Che, Yuanzhen Li

**Affiliations:** ^1^Department of Internal Medicine Nursing, School of Nursing, Wannan Medical College, 22 Wenchang West Road, Higher Education Park, Wuhu City, Anhui Province, China; ^2^Obstetrics and Gynecology Nursing, School of Nursing, Wannan Medical College, 22 Wenchang West Road, Higher Education Park, Wuhu City, Anhui Province, China; ^3^Department of Pediatric Nursing, School of Nursing, Wannan Medical College, 22 Wenchang West Road, Higher Education Park, Wuhu City, Anhui Province, China; ^4^Department of Surgical Nursing, School of Nursing, Wannan Medical College, 22 Wenchang West Road, Higher Education Park, Wuhu City, Anhui Province, China; ^5^Department of Emergency and Critical Care Nursing, School of Nursing, Wannan Medical College, 22 Wenchang West Road, Higher Education Park, Wuhu City, Anhui Province, China; ^6^Rehabilitation Nursing, School of Nursing, Wannan Medical College, 22 Wenchang West Road, Higher Education Park, Wuhu City, Anhui Province, China; ^7^Department of Nursing, Yijishan Hospital, The First Affiliated Hospital of Wannan Medical College, Zheshan West Road, Yijishan District, Wuhu City, Anhui Province, China

## Abstract

**Objectives:**

Undernutrition early in life may increase the incidence of adverse effects on adult health. The relations between undernutrition and obesity parameters (body mass index (BMI) and WC (waist circle)) and hypertension were often contradictory. Our study is aimed at identifying the combined effects of famine exposure and obesity parameters on hypertension in middle-aged and older Chinese.

**Design:**

A population-based cross-sectional study. *Setting*. Data were selected from the China Health and Retirement Longitudinal Study Wave2011 (CHARLS Wave2011). *Participants*. The sample included 12945 individuals aged 45 to 96. *Main Outcome Measurements*. The study analyzed data from 12945 middle-aged and older Chinese selected from CHARLS Wave2011. Differences between baseline characteristics and famine exposure/BMI levels/WC levels were evaluated using the *t*-, Chi-square- (*χ*^2^-), and *F*-test. Then, the difference in the prevalence of hypertension between baseline characteristics was estimated by the *t*- and *χ*^2^-test. Finally, multivariable-adjusted logistic regression models were used to explore the associations of famine exposure and obesity parameters with odds of prevalence of hypertension.

**Results:**

Among the 12945 participants, 1548 (11.96%) participants had been exposed to the Chinese famine during the fetal group, whereas 5101 (39.41%) participants and 4362 (33.70%) participants had been exposed to the famine during childhood and adolescence/adult group, respectively. Regarding the participants with BMI levels, 3746 (28.94%) were overweight, and 1465 (11.32%) were obese, whereas 5345 (41.29%) of the participants with WC levels were obese, respectively. Furthermore, 1920 (31.17%) had hypertension in males and 2233 (32.91%) in females. In multivariable-adjusted models, famine exposure and obesity parameters were related with prevalence of hypertension independently in total populations ((1) model three^c^, famine exposure with prevalence of hypertension: the fatal-exposed vs. no-exposed group (OR1.27; 95% CI 1.08, 1.49); childhood-exposed vs. no-exposed group (OR1.64; 95% CI 1.44, 1.87); the adolescence/adult-exposed vs. no-exposed group (OR3.06; 95% CI 2.68, 3.50); *P* for trend < 0.001; (2) model three^e^, famine exposure with prevalence of hypertension: the fatal-exposed vs. no-exposed group (OR1.25; 95% CI 1.06, 1.47); childhood-exposed vs. no-exposed group (OR1.52; 95% CI 1.34, 1.73); the adolescence/adult-exposed vs. no-exposed group (OR2.66; 95% CI 2.33, 3.03); *P* for trend < 0.001; (3) model three^g^, BMI levels with prevalence of hypertension: overweight vs. normal (OR1.75; 95% CI 1.60, 1.91); obesity vs. normal (OR2.79; 95% CI 2.48, 3.15); *P* for trend < 0.001; (4) WC levels with prevalence of hypertension: overweight vs. normal (OR1.42; 95% CI 1.36, 1.48)). When stratified by sex, results in both males and females were mostly similar to those in the total population. In general, interaction analysis in the multivariable-adjusted model, compared with the combination of normal BMI/WC levels and no-exposed famine group, all groups trended towards higher odds of prevalence of hypertension (the greatest increase in odds, adolescence/adult-exposed group with obesity in BMI levels: (OR8.13; 95% CI 6.18, 10.71); adolescence/adult-exposed group with obesity in WC levels: (OR6.36; 95% CI 5.22, 7.75); *P* for interaction < 0.001). When stratified by sex, the results in both males and females were also similar to those in the total population.

**Conclusion:**

Our data support a strongly positive combined effect of famine exposure and obesity parameters on hypertension in middle-aged and elderly Chinese.

## 1. Introduction

Hypertension or elevated blood pressure (BP) is a severe medical condition that significantly increases the risks of cardiovascular diseases (CVD) as well as other chronic diseases [1–3], such as congenital heart disease, heart failure, heart attack, peripheral vascular disease, stroke, and vascular disease. Hypertension modifiable risk factors [4–8] include age, sex, life stress, excessive drinking, high-salt diet, being overweight or obese, saturated fat and trans fats, tobacco use, low intake of fruits and vegetables, lack of physical activity, family history, low diet in vitamin D, advanced age, and coexisting diseases. Though the etiology of hypertension is complex, it was known as one of the strongest risk factors was overweight or obesity. Thus, increased body mass index (BMI) or centrally located body fat (especially waist circle (WC)) increases the risk of hypertension. In addition to known and probable risk factors for hypertension, early life malnutrition may also have an effect on hypertension.

It was hypothesized that early developmental adaptions in response to malnutrition in early life, which are the main factor for short-term survival, have adverse cardiovascular outcomes [9, 10]. Historical famine exposure has provided a unique and natural opportunity to identify the hypothesis. Several previous studies [11–23] have provided evidence to support the relationship between famine exposure and increased risk of hypertension. Most studies [11, 13, 14, 16–23] have found that exposure to famine in early life could increase the risk of hypertension/BP in adulthood. Furthermore, exposure to famine has more deleterious effects on adult health for females than males [12, 15]. However, other studies [13, 24, 25] found no relationship between famine exposure and hypertension. Therefore, the relationship between famine exposure in early life and the risk of hypertension/BP needs to be further investigated. Moreover, studies also provided that malnutrition in early life [26–31] was more positively correlated with obesity among adults in late life. Generally speaking, it is not completed understood association and interaction analysis between famine exposure and obesity parameters (BMI and WC) and hypertension in the midage and older adult.

Given the limitations of previous studies, our study analyzed data from the China Health and Retirement Longitudinal Study Wave2011 (CHARLS Wave2011) and is aimed at exploring the individual and combined effects of famine exposure and obesity parameters on hypertension after adjustment for potential confounding variables.

## 2. Methods

### 2.1. Study Design and Setting

Data from the China Health and Retirement Longitudinal Study Wave2011 (CHARLS Wave2011) were used in our study. The CHARLS was a nationally representative longitudinal study conducted by the China Centre for Economic Research at Peking University [32]. In the CHARLS Wave2011, 13107 individuals were recruited for the baseline, after excluding participants with missing data, 12945 individuals were included in our study. All data are openly published as microdata at http://charls.pku.edu.cn/index/zh-cn.html with no direct contact with individuals. The Ethics Committee of the China Centre for Economic Research at Peking University approved the study; all individuals have provided informed consent before the data collection.

### 2.2. Individuals

The individuals of the study were selected from the CHARLS Wave2011 [32]. The mean age of CHARLS involved 12945 individuals was 59.33 years (standard deviation (SD) = 9.48, ranged from 45 to 96 years). The mean age was 59.88 years (SD = 9.36, ranged from 45 to 90 years) in males and 58.83 years (SD = 9.55, ranged from 45 to 96 years) in females.

### 2.3. Baseline Characteristics

Baseline characteristics including age, sex (0 = male; 1 = female), marital status (0 = single; 1 = married), education (0 = illiterate; 1 = less than elementary school; 2 = high school; 3 = above vocational school), living place (0 = rural; 1 = urban), smoking status (0 = no; 1 = former smoke; 2 = current smoke), drinking status (0 = no; 1 = less than once a month; 2 = more than once a month), eating habit (0 = ≤2 meals per day; 1 = 3 meals per day; 2 = ≥4 meals per day), social activities (0 = no; 1 = yes), experience of traumatic events (0 = no; 1 = yes), and physical exercise habit (0 = no; 1 = less than regular physical exercises; 2 = regular physical exercises) were collected by self-report. Most variables were depending on our previous research studies [33–38].

### 2.4. Measurements

BMI was calculated based on the measured weight and height of the participants. Tapeline was localized at navel levels to read the WC at the end of exhalation. Using the standard China definition, BMI was categorized into three groups [39]: obesity (BMI ≥ 28 kg/m^2^), overweight (24 ≤ BMI < 28 kg/m^2^), and underweight and normal (BMI < 24 kg/m^2^). Central obesity was defined as a WC [40] of ≥85 cm for females and ≥90 cm for males. Hypertension was defined as systolic blood pressure (SBP) of ≥140 mmHg and/or diastolic blood pressure (DBP) of ≥90 mmHg; the definition has been used in our previous studies [33, 35, 37, 38].

### 2.5. Exposure Age and Exposed Groups

Famine exposure is set up on the previous Chinese famine study [41]; famine exposure was categorized into four exposure groups: no-exposed group (birth year between 1963-01-01 and 1966-12-31), fetal-exposed group (birth year 1959-01-01 and 1962-12-31), childhood-exposed group (birth year 1949-01-01 and 1958-12-31), and adolescence/adult-exposed group (birth year between1921-01-01 and 1948-12-31).

### 2.6. Statistical Analysis

Analyses were conducted using SPSS software, version 22.0 (IBM SPSS, Armonk, NY, USA). The data are presented as mean ± SD unless indicated otherwise. Means and SD (continuous data) were used to measure the continuous variable (age), and count and percentage were used to describe categorical variables (sex, education, marital status, living place, drinking status, smoking habit, eating habit, social activities, the experience of traumatic events, taking physical activity or exercise, famine exposure, BMI levels, WC levels, and hypertension categories). Between-group differences according to hypertension (hypertension and no-hypertension) were evaluated by the chi-square test (categorical data). Differences between baseline characteristics (sex, education, marital status, living place, drinking status, smoking habit, eating habit, social activities, the experience of traumatic events, and taking physical activity or exercise) and categories of famine exposure groups/BMI levels/WC levels were also evaluated using the chi-square test (categorical data). Age between groups was used by *t*- or *F*-test. Logistic regression models were used to compute ORs with accompanying 95% CIs as estimates of associations of BMI/WC levels and exposure groups separately and in combination, with the prevalence of hypertension. Two-tailed *P* < 5% was considered to indicate statistical significance.

## 3. Results

Table 1 shows the basic characteristics of participants. A total of 12945 individuals were enrolled into the study; 6159 (47.58%) participants and 6786 (52.42%) participants were male and female, respectively. Among males, 676 (10.98%) participants had been exposed to the Chinese famine during the fetal group, whereas 2448 (39.75%) participants and 2233 (36.26%) participants had been exposed to the famine during childhood and adolescence/adult groups, respectively. Among females, 872 (12.85%) participants had been exposed to the Chinese famine during the fetal group, whereas 2653 (39.10%) participants and 2129 (31.37%) participants had been exposed to the famine during childhood and adolescence/adult groups, respectively. The distribution of living place and experience of traumatic events did not demonstrate significantly statistical differences among the four birth groups. On the other hand, the difference was observed in the distribution of age, sex, education, marital status, smoking status, drinking status, eating habit, social events, and physical exercise habit. Regarding the males, 4088 (66.37%) were underweight and normal, 1572 (25.52%) were overweight, and 499 (8.10%) were obese, whereas 3646 (53.73%), 2174 (32.04%), and 966 (14.24%) of the females were underweight and normal, overweight, and obese, respectively. Furthermore, significant differences in distribution were observed between BMI levels in all variables, including age, sex, education, marital status, living place, smoking status, drinking status, eating habit, social events, the experience of traumatic events, and physical exercise habit. Among the WC measures, 1839 (29.86%) were central obesity in males and 3506 (51.67%) in females. The proportions on the characteristics were statistically different between the WC groups except for age and marital status.

Table 2 shows the characteristics of study participants categorized by blood pressure status. Of the participants, 1920 (31.17%) reported having hypertension in male and 2233 (32.91%) in the female. Significant differences were observed in age, sex, education, marital status, living place, drinking status, the experience of traumatic events, famine groups, BMI levels, and WC groups (*P* < 0.05) between participants with and without hypertension.

Table 3 shows the separate associations of famine exposure, BMI, and central obesity with the prevalence of hypertension. Firstly, after controlling for confounding factors including age, education, marital status, living place, smoking status, drinking status, eating habit, social activities, the experience of traumatic events, taking physical activity or exercise, and famine exposure in a multivariable logistic regression model three, higher odds of prevalence of hypertension in the total population were observed with increasing levels of BMI (overweight vs. normal: 1.75 (95% CI 1.60, 1.91); obesity vs. normal: 2.79 (95% CI 2.48, 3.15)) and WC (overweight vs. normal: 1.42 (95% CI 1.36, 1.48)) independently of famine groups only (BMI, *P* for trend < 0.001). When stratified by sex, the results of model three in both males and females were mostly similar to those in the total population. Secondly, after controlling for confounding factors including age, education, marital status, living place, smoking status, drinking status, eating habit, social activities, the experience of traumatic events, taking physical activity or exercise, and BMI in a multivariable logistic regression model three, higher odds of prevalence of hypertension in the total population were observed with famine-exposed groups (fatal-exposed group vs. nonexposed group: 1.27 (95% CI 1.08, 1.49); childhood-exposed group vs. nonexposed group: 1.64 (95% CI 1.44, 1.87); adolescence/adult-exposed group vs. nonexposed group: 3.06 (95% CI 2.68, 3.50), *P* for trend < 0.001) independently of BMI only (*P* for trend < 0.001). When stratified by sex, the results of model three in both males and females were mostly similar to those in the total population. Lastly, after controlling for confounding factors including age, education, marital status, living place, smoking status, drinking status, eating habit, social activities, the experience of traumatic events, taking physical activity or exercise, and WC in a multivariable logistic regression model three, higher odds of prevalence of hypertension in the total population were observed with famine-exposed groups (fatal-exposed group vs. nonexposed group: 1.25 (95% CI 1.06, 1.47); childhood-exposed group vs. nonexposed group: 1.52 (95% CI 1.34, 1.73); adolescence/adult-exposed group vs. nonexposed group: 2.66 (95% CI 2.33, 3.03), *P* for trend < 0.001) independently of WC only (*P* for trend < 0.001). When stratified by sex, the results of model three in both males and females were mostly similar to those in the total population.

Table 4 shows the combined associations of obesity parameters and famine exposure with the prevalence of hypertension in males. Compared with the combination of the normal BMI/WC level and no-exposed famine group, all groups trended towards higher odds of prevalence of hypertension except the obesity; furthermore, in multivariable model one, the greatest increase in odds was observed for the adolescence/adult-exposed group and obesity combination (adolescence/adult-exposed group and obesity in BMI: OR 7.38; 95% CI 4.81, 11.32; adolescence/adult-exposed group and obesity in WC: OR 6.13; 95% CI 4.54, 8.26). And similarly, in multivariable-adjusted model two, the highest odds of prevalence of hypertension were observed for the adolescence/adult exposed group and obesity combination (adolescence/adult-exposed group and obesity in BMI: OR 6.87; 95% CI 4.47, 10.57; adolescence/adult-exposed group and obesity in WC: OR 5.75; 95% CI 4.26, 7.77). Additionally, in multivariable-adjusted model three, the highest odds of prevalence of hypertension were observed for the adolescence/adult-exposed group and obesity combination (adolescence/adult-exposed group and obesity in BMI: OR 7.30; 95% CI 4.74, 11.25; adolescence/adult-exposed group and obesity in WC: OR 6.68; 95% CI 4.92, 9.07). Finally, combined associations of obesity parameters and famine exposure with the prevalence of hypertension were observed in males (*P*interaction = <0.001).

Table 5 shows the combined associations of obesity parameters and famine exposure with the prevalence of hypertension in females. Compared with the combination of the normal BMI/WC level and no-exposed famine group, all groups trended towards higher odds of prevalence of hypertension; furthermore, in multivariable model one, the greatest increase in odds was observed for the adolescence/adult-exposed group and obesity combination (adolescence/adult-exposed group and obesity in BMI: OR 10.38; 95% CI 7.26, 14.48; adolescence/adult-exposed group and obesity in WC: OR 7.59; 95% CI 5.86, 9.84). And similarly, in multivariable-adjusted model two, the highest odds of prevalence of hypertension were observed for the adolescence/adult-exposed group and obesity combination (adolescence/adult-exposed group and obesity in BMI: OR 8.88; 95% CI 6.18, 12.75; adolescence/adult-exposed group and obesity in WC: OR 6.58; 95% CI 5.05, 8.58). Additionally, in multivariable-adjusted model three, the highest odds of prevalence of hypertension were observed for the adolescence/adult-exposed group and obesity combination (adolescence/adult-exposed group and obesity in BMI: OR 8.89; 95% CI 6.19, 12.78; adolescence/adult-exposed group and obesity in WC: OR 6.59; 95% CI 5.05, 8.59). Finally, combined associations of obesity parameters and famine exposure with the prevalence of hypertension were observed in females (*P*interaction < 0.001).

Table 6 shows the combined associations of obesity parameters and famine exposure with the prevalence of hypertension in the total population. Compared with the combination of the normal BMI/WC level and no-exposed famine group, all groups trended towards higher odds of prevalence of hypertension; furthermore, in multivariable model one, the greatest increase in odds was observed for the adolescence/adult-exposed group and obesity combination (adolescence/adult-exposed group and obesity in BMI: OR 9.04; 95% CI 6.89, 11.86; adolescence/adult-exposed group and obesity in WC: OR 7.05; 95% CI 5.80, 8.56). And similarly, in multivariable-adjusted model two, the highest odds of prevalence of hypertension were observed for the adolescence/adult-exposed group and obesity combination (adolescence/adult-exposed group and obesity in BMI: OR 7.94; 95% CI 6.03, 10.44; adolescence/adult-exposed group and obesity in WC: OR 6.29; 95% CI 5.16, 7.66). Additionally, in multivariable-adjusted model three, the highest odds of prevalence of hypertension were observed for the adolescence/adult-exposed group and obesity combination (adolescence/adult-exposed group and obesity in BMI: OR 8.13; 95% CI 6.18, 10.71; adolescence/adult-exposed group and obesity in WC: OR 6.36; 95% CI 5.22, 7.75). Finally, combined associations of obesity parameters and famine exposure with the prevalence of hypertension were observed in the total population (*P*interaction < 0.001).

## 4. Discussion

In the study, we found that the individuals who had been exposed to famine in early life had an increased risk of hypertension in adults. After adjustment for the full set of potential confounders, including age, education, marital status, living place, smoking status, drinking status, eating habit, social activities, the experience of traumatic events, taking physical activity or exercise, and obesity parameters (BMI or WC), the associations still can be found in males and females. Additionally, our study found that there were linear trends in the associations of BMI with hypertension. After adjustment for observed potential confounders, the associations still existed both in males and females. In summary, our study supports a strongly positive combined effect of famine exposure and obesity parameters on hypertension in middle-aged and elderly Chinese. When stratified by sex, similar results were found with respect to the association.

The Chinese famine of 1959–61 caused over 30 million excess deaths [42]. A large number of such studies have explored the associations of famine exposure during early life with the risk of hypertension in adults, and there were no consistent associations observed for these studies. Therefore, our study attempted to explore the associations between obesity parameters (BMI or WC) and hypertension based on a national study from CHARLS2011. In conclusion, the findings from our study support a strongly positive combined effect of famine exposure and obesity parameters (BMI or WC) on hypertension in middle-aged and elderly Chinese. Both nutrition intervention for exposure to the famine in early life and weight control in later life may be required to substantially reduce the risk of hypertension in later life.

The effect of the worst famine to hypertension may be masked, however, by a selection effect of survivors who might be healthier than the frail members more likely to survive. The finding is in line with Darwin's theory of survival of the fittest [43]. Individuals who were exposed to famine in early life should decrease the risk of hypertension in adults. However, this was not observed in our research. The reason for the inconsistency may be due to the environmental changes. When facing the later “rich” environment, the risk of hypertension may be increased.

Our results are partly in line with several previous studies. Although the Dutch famine and the Leningrad siege study [44–46] have generally agreed that early-life exposure to famine was not associated with hypertension, most current published research findings [11, 12, 14–23] in China indicated that exposure to famine in early life increased the risk of hypertension. However, it was found there was no association between the Chinese famine and hypertension risk in Chongqing [24]. Such discrepancies between these studies may be a result of methodological differences in definitions of the different sample selection effect and famine exposure groups. Additionally, these studies have been criticized for not being adjusted to the confounding bias of age. To control the age confounding, we categorized the famine exposure into four exposure groups based on the birth year and we also combined the no-exposure as the reference group to identify the effect of the fetal-exposed group, childhood-exposed group, and adolescence/adult-exposed group. Our study found that early famine exposure was associated with an increased risk of hypertension. The sex difference of early life famine exposure and hypertension were common in other studies [15, 17]. Furthermore, exposure to famine during early life exerted more deleterious effects on females than males. This could be explained by the fact the female may suffer more than males during early life, because of the dominance of a patriarchal mentality in China [47]. The potential mechanisms of the associations between famine exposure in early life and the increased risk of hypertension in later life were still not fully understood. Animal experiments [48, 49] have proved that malnutrition in early life could result in elevated BP in later life. Additionally, epigenetic might play a role in the association between famine exposure in early life and hypertension in late life [50, 51].

In our research, participants who were overweight/obese and exposed to famine in adolescence/adult tended to have a higher risk of hypertension. The results indicated the good nutrition in adults did not match poor nutrition in early life, which might elevate the relative risk of hypertension in later life [52]. Furthermore, our data support a strongly positive combined effect of famine exposure and obesity parameters on hypertension in middle-aged and elderly Chinese. However, the previous studies focused on the relationship between famine exposure and health outcomes in late adolescence and adulthood. Most of the previous studies meant exactly that famine exposure was at a higher risk for health outcomes in late adolescence and adulthood. Exposure to Chinese famine in early life was related to increased risk of metabolic syndrome [41, 44, 53–57], weight gain [26–31], diabetes [58–73], hypertension [11, 12, 14–23], cognitive decline [74–80], and depressive syndrome [42, 76, 81, 82]. In addition, our study found that there were linear trends in the associations of BMI with hypertension which was consistent with our previous study [83]. However, several studies proved that there were different associations of body mass index with health outcomes, such as U- [84–88], J- [89–95], and reverse J-shape [96, 97]. A U- or a J-shaped association between BMI and cardiovascular events is often described. This U-shaped association may result from the effect of medication use or unintentional weight loss. By contrast, patients with other severe heart diseases or undergoing cardiac surgery presented a reverse J-shape suggesting the low body mass index associated with the highest mortality [98].

Though so many studies have explored the association analysis between famine exposure/obesity parameters and BP, there were only two studies that explored the combined effect of obesity parameters on the relation between famine exposure and hypertension. Yu et al. [19] found that interactions between famine and obesity on hypertension prevalence risk were not observed. In contrast, Li et al. [11] reported that a stronger interaction between obesity and famine exposure with regard to BP among individuals who were exposed to famine during fetal life and had a western dietary pattern in adults was observed. Interestingly, our data support a strongly positive combined effect of famine exposure and obesity parameters on hypertension in middle-aged and elderly Chinese. The difference between our research and others may be due to the different populations, different definitions of famine exposure cohort, and different confounding variables by controlling. The individuals in our study were midaged and elderly Chinese, where the mean age at recruitment was older than in Yu et al.' s study, and the level of socioeconomic development also made some contribution to ontogenetic development. In addition, the participants were similar in China and its socioeconomic background, and this phenomenon could be explained by the cumulative effect.

Several limitations have to be taken into account as well. Firstly, selection bias was to be considered: famine may weed out the frail members and leave the healthier ones. Secondly, individual famine exposure data have not been collected. Lastly, not all families were equally affected by famine exposure. However, our study provided a large data that could be explored further in the combined effect of famine exposure and obesity parameters (BMI or WC) on hypertension. Moreover, a significant strength of the study is the large sample of 12945 middle-aged and older Chinese. Another strength is the analytical method of controlling for a number of confounders.

## 5. Conclusions

Our data support a strongly positive combined effect of famine exposure and obesity parameters on hypertension in middle-aged and elderly Chinese. Both nutrition intervention for exposure to the famine in early life and weight reduction in later life may be required to substantially reduce the risk of hypertension in later life.

## Figures and Tables

**Table 1:** Characteristics of participants in the cross-sectional study by level of famine exposure, BMI, and central obesity (*N* = 12945).

Characteristics	Famine exposure				*χ*^2^/*F*	*P*	BMI			*χ*^2^/*F*	*P*	Central obesity		*χ*^2^/*t*	*P*
	No-exposed	Fetal-exposed	Childhood-exposed	Adolescence/adult-exposed			Underweight and normal	Overweight	Obesity			Normal	Obesity		
*N*	1934	1548	5101	4362			7734	3746	1465			7600	5345		
Age	46.75 ± 1.07	50.26 ± 1.17	57.54 ± 2.78	70.22 ± 5.90	21351.166	<0.001	60.38 ± 9.78	57.88 ± 8.77	57.47 ± 8.78	121.799	<0.001	59.45 ± 9.57	59.15 ± 9.35	1.773	0.076
Sex															
Male	802 (41.47)	676 (43.67)	2448 (47.99)	2233 (51.19)	61.618	<0.001	4088 (52.86)	1572 (41.96)	499 (34.06)	241.067	<0.001	4320 (56.84)	1839 (34.41)	633.337	<0.001
Female	1132 (58.53)	872 (56.33)	2653 (52.01)	2129 (48.81)			3646 (47.14)	2174 (58.04)	966 (65.94)			3280 (43.16)	3506 (65.59)		
Education															
Illiterate	210 (10.86)	263 (16.99)	1442 (28.27)	1689 (38.72)	1102.252	<0.001	2282 (29.51)	933 (24.91)	389 (26.55)	75.386	<0.001	2037 (26.8)	1567 (29.32)	29.604	<0.001
Less than elementary school	1452 (75.08)	926 (59.82)	3163 (62.01)	2398 (54.97)			4742 (61.31)	2296 (61.29)	901 (61.50)			4776 (62.84)	3163 (59.18)		
High school	190 (9.82)	293 (18.93)	364 (7.14)	63 (1.44)			477 (6.17)	326 (8.70)	107 (7.30)			541 (7.12)	369 (6.9)		
Above vocational school	82 (4.24)	66 (4.26)	132 (2.59)	212 (4.86)			233 (3.01)	191 (5.10)	68 (4.64)			246 (3.24)	246 (4.6)		
Marital status															
Single	68 (3.52)	93 (6.01)	427 (8.37)	1065 (24.42)	831.933	<0.001	1148 (14.84)	356 (9.50)	149 (10.17)	74.624	<0.001	986 (12.97)	667 (12.48)	0.690	0.406
Married	1866 (96.48)	1455 (93.99)	4674 (91.63)	3297 (75.58)			6586 (85.16)	3390 (90.50)	1316 (89.83)			6614 (87.03)	4678 (87.52)		
Living place															
Rural	1178 (60.91)	961 (62.08)	3228 (63.28)	2790 (63.96)	6.090	0.107	5299 (68.52)	2103 (56.14)	755 (51.54)	259.203	<0.001	5218 (68.66)	2939 (54.99)	251.674	<0.001
Urban	756 (39.09)	587 (37.92)	1873 (36.72)	1572 (36.04)			2435 (31.48)	1643 (43.86)	710 (48.46)			2382 (31.34)	2406 (45.01)		
Smoking status															
No	1302 (67.32)	981 (63.37)	2998 (58.77)	2467 (56.56)	174.199	<0.001	4209 (54.42)	2479 (66.18)	1060 (72.35)	359.354	<0.001	4002 (52.66)	3746 (70.08)	495.644	<0.001
Former smoker	111 (5.74)	76 (4.91)	426 (8.35)	564 (12.93)			647 (8.37)	383 (10.22)	147 (10.03)			667 (8.78)	510 (9.54)		
Current smoker	521 (26.94)	491 (31.72)	1677 (32.88)	1331 (30.51)			2878 (37.21)	884 (23.6)	258 (17.61)			2931 (38.57)	1089 (20.37)		
Drinking status															
No	1272 (65.77)	1001 (64.66)	3369 (66.05)	3042 (69.74)	35.519	<0.001	4963 (64.17)	2620 (69.94)	1101 (75.15)	94.448	<0.001	4751 (62.51)	3933 (73.58)	180.725	<0.001
Less than once a month	179 (9.26)	158 (10.21)	405 (7.94)	292 (6.69)			640 (8.28)	285 (7.61)	109 (7.44)			656 (8.63)	378 (7.07)		
More than once a month	483 (24.97)	389 (25.13)	1327 (26.01)	1028 (23.57)			2131 (27.55)	841 (22.45)	255 (17.41)			2193 (28.86)	1034 (19.35)		
Eating habit															
≤2 meals per day	272 (14.06)	203 (13.11)	585 (11.47)	652 (14.95)	37.603	<0.001	1157 (14.96)	407 (10.86)	148 (10.10)	73.602	<0.001	1101 (14.49)	611 (11.43)	39.126	<0.001
3 meals per day	1643 (84.95)	1328 (85.79)	4414 (86.53)	3642 (83.49)			6425 (83.07)	3294 (87.93)	1308 (89.28)			6354 (83.61)	4673 (87.43)		
≥4 meals per day	19 (0.98)	17 (1.10)	102 (2)	68 (1.56)			152 (1.97)	45 (1.20)	9 (0.61)			145 (1.91)	61 (1.14)		
Social events															
No	844 (43.64)	683 (44.12)	2597 (50.91)	2313 (53.03)	69.975	<0.001	4085 (52.82)	1715 (45.78)	637 (43.48)	75.751	<0.001	3931 (51.72)	2506 (46.88)	29.390	<0.001
Yes	1090 (56.36)	865 (55.88)	2504 (49.09)	2049 (46.97)			3649 (47.18)	2031 (54.22)	828 (56.52)			3669 (48.28)	2839 (53.12)		
Experience of traumatic events															
No	1743 (90.12)	1396 (90.18)	4579 (89.77)	3959 (90.76)	2.651	0.449	6947 (89.82)	3379 (90.20)	1351 (92.22)	7.991	0.018	6798 (89.45)	4879 (91.28)	11.948	0.001
Yes	191 (9.88)	152 (9.82)	522 (10.23)	403 (9.24)			787 (10.18)	367 (9.80)	114 (7.78)			802 (10.55)	466 (8.72)		
Physical exercise habit															
No physical exercise	1187 (61.38)	919 (59.37)	3132 (61.40)	2793 (64.03)	18.363	0.005	4806 (62.14)	2293 (61.21)	932 (63.62)	13.830	0.008	4710 (61.97)	3321 (62.13)	6.259	0.044
Less than regular physical exercises	389 (20.11)	321 (20.74)	973 (19.07)	745 (17.08)			1504 (19.45)	679 (18.13)	245 (16.72)			1471 (19.36)	957 (17.90)		
Regular physical exercises	358 (18.51)	308 (19.90)	996 (19.53)	824 (18.89)			1424 (18.41)	774 (20.66)	288 (19.66)			1419 (18.67)	1067 (19.96)		

**Table 2:** Characteristics of study participants of cross-sectional study categorized by blood pressure status (*N* = 12945).

Variables	Without hypertension *N* = 8792	Hypertension *N* = 4153	Total	*χ*^2^/*t*	*P*
Age	58.07 ± 8.99	62.00 ± 9.92	59.33 ± 9.48	-21.720	<0.001
Sex				4.445	0.035
Male	4239 (48.21)	1920 (46.23)	6159 (47.58)		
Female	4553 (51.79)	2233 (53.77)	6786 (52.42)		
Education					
Illiterate	2262 (25.73)	1342 (32.31)	3604 (27.84)	69.641	<0.001
Less than elementary school	5526 (62.85)	2413 (58.1)	7939 (61.33)		
High school	673 (7.65)	237 (5.71)	910 (7.03)		
Above vocational school	331 (3.76)	161 (3.88)	492 (3.8)		
Marital status					
Single	919 (10.45)	734 (17.67)	1653 (12.77)		<0.001
Married	7873 (89.55)	3419 (82.33)	11292 (87.23)	132.050	
Living place					
Rural	5671 (64.5)	2486 (59.86)	8157 (63.01)	26.072	<0.001
Urban	3121 (35.5)	1667 (40.14)	4788 (36.99)		
Smoking status					
No	5265 (59.88)	2483 (59.79)	7748 (59.85)	4.187	0.123
Former smoke	770 (8.76)	407 (9.80)	1177 (9.09)		
Current smoke	2757 (31.36)	1263 (30.41)	4020 (31.05)		
Drinking status					
No	5852 (66.56)	2832 (68.19)	8684 (67.08)	11.233	0.004
Less than once a month	750 (8.53)	284 (6.84)	1034 (7.99)		
More than once a month	2190 (24.91)	1037 (24.97)	3227 (24.93)		
Eating habit					
≤2 meals per day	1144 (13.01)	568 (13.68)	1712 (13.23)	1.258	0.533
3 meals per day	7505 (85.36)	3522 (84.81)	11027 (85.18)		
≥4 meals per day	143 (1.63)	63 (1.52)	206 (1.59)		
Social events					
No	4336 (49.32)	2101 (50.59)	6437 (49.73)	1.827	0.177
Yes	4456 (50.68)	2052 (49.41)	6508 (50.27)		
Experience of traumatic events					
No	7881 (89.64)	3796 (91.40)	11677 (90.20)	9.950	0.002
Yes	911 (10.36)	357 (8.60)	1268 (9.80)		
Physical exercise habit					
No physical exercise	5409 (61.52)	2622 (63.14)	8031 (62.04)	3.162	0.206
Less than regular physical exercises	1675 (19.05)	753 (18.13)	2428 (18.76)		
Regular physical exercises	1708 (19.43)	778 (18.73)	2486 (19.2)		
Famine exposure					
No-exposed	1536 (17.47)	398 (9.58)	1934 (14.94)	420.894	<0.001
Fetal-exposed	1167 (13.27)	381 (9.17)	1548 (11.96)		
Childhood-exposed	3609 (41.05)	1492 (35.93)	5101 (39.41)		
Adolescence/adult-exposed	2480 (28.21)	1882 (45.32)	4362 (33.7)		
BMI					
Underweight and normal	5625 (63.98)	2109 (50.78)	7734 (59.75)	257.301	<0.001
Overweight	2387 (27.15)	1359 (32.72)	3746 (28.94)		
Obesity	780 (8.87)	685 (16.49)	1465 (11.32)		
Central obesity					
Normal	5647 (64.23)	1953 (47.03)	7600 (58.71)	344.333	<0.001
Obesity	3145 (35.77)	2200 (52.97)	5345 (41.29)		

**Table 3:** Separate associations of famine exposure, BMI, and central obesity with the prevalence of hypertension (*N* = 12945).

Variables	Male (OR and 95% CI for hypertension)			Female (OR and 95% CI for hypertension)			Total (OR and 95% CI for hypertension)		
Famine exposure	Model one^a^	Model two^b^	Model three^c^	Model one^a^	Model two^b^	Model three^c^	Model one^a^	Model two^b^	Model three^c^
								
No-exposed	1.00 (reference)	1.00 (reference)	1.00 (reference)	1.00 (reference)	1.00 (reference)	1.00 (reference)	1.00 (reference)	1.00 (reference)	1.00 (reference)
Fetal-exposed	1.28 (1.01, 1.63)	1.33 (1.04, 1.69)	1.31 (1.03, 1.67)	1.24 (1.00, 1.53)	1.22 (0.98, 1.51)	1.23 (0.99, 1.53)	1.26 (1.07, 1.48)	1.27 (1.08, 1.49)	1.27 (1.08, 1.49)
Childhood-exposed	1.47 (1.22, 1.78)	1.59 (1.32, 1.93)	1.59 (1.31, 1.93)	1.69 (1.43, 2.00)	1.66 (1.40, 1.97)	1.67 (1.41, 1.99)	1.60 (1.41, 1.81)	1.65 (1.45, 1.88)	1.64 (1.44, 1.87)
Adolescence/adult-exposed	2.18 (1.80, 2.63)	2.46 (2.02, 2.98)	2.52 (2.07, 3.07)	3.87 (3.27, 4.59)	3.82 (3.19, 4.59)	3.83 (3.19, 4.60)	2.93 (2.58, 3.32)	3.09 (2.71, 3.53)	3.06 (2.68, 3.50)
*P* for trend	<0.001	<0.001	<0.001	<0.001	<0.001	<0.001	<0.001	<0.001	<0.001
Famine exposure		Model two^d^	Model three^e^		Model two^d^	Model three^e^		Model two^d^	Model three^e^
No-exposed		1.00 (reference)	1.00 (reference)		1.00 (reference)	1.00 (reference)		1.00 (reference)	1.00 (reference)
Fetal-exposed		1.30 (1.02, 1.66)	1.28 (1.01, 1.64)		1.20 (0.96, 1.49)	1.21 (0.97, 1.50)		1.25 (1.06, 1.47)	1.25 (1.06, 1.47)
Childhood-exposed		1.52 (1.26, 1.85)	1.51 (1.25, 1.84)		1.52 (1.28, 1.81)	1.53 (1.29, 1.82)		1.53 (1.34, 1.74)	1.52 (1.34, 1.73)
Adolescence/adult-exposed		2.24 (1.85, 2.72)	2.28 (1.88, 2.77)		3.23 (2.69, 3.87)	3.24 (2.70, 3.89)		2.68 (2.35, 3.05)	2.66 (2.33, 3.03)
*P* for trend		<0.001	<0.001		<0.001	<0.001		<0.001	<0.001
BMI	Model one^a^	Model two^f^	Model three^g^	Model one^a^	Model two^f^	Model three^g^	Model one^a^	Model two^f^	Model three^g^
Underweight and normal	1.00 (reference)	1.00 (reference)	1.00 (reference)	1.00 (reference)	1.00 (reference)	1.00 (reference)	1.00 (reference)	1.00 (reference)	1.00 (reference)
Overweight	1.68 (1.49, 1.90)	1.83 (1.61, 2.08)	1.88 (1.66, 2.14)	1.39 (1.24, 1.56)	1.61 (1.43, 1.82)	1.62 (1.44, 1.82)	1.52 (1.40, 1.65)	1.71 (1.57, 1.86)	1.75 (1.60, 1.91)
Obesity	2.47 (2.05, 2.99)	2.78 (2.29, 3.38)	2.88 (2.36, 3.50)	2.23 (1.93, 2.58)	2.68 (2.30, 3.12)	2.67 (2.29, 3.12)	2.34 (2.09, 2.63)	2.72 (2.41, 3.06)	2.79 (2.48, 3.15)
*P* for trend	<0.001	<0.001	<0.001	<0.001	<0.001	<0.001	<0.001	<0.001	<0.001
Central obesity	Model one^a^	Model two^f^	Model three^g^	Model one^a^	Model two^f^	Model three^g^	Model one^a^	Model two^f^	Model three^g^
Normal	1.00(reference)	1.00 (reference)	1.00 (reference)	1.00 (reference)	1.00 (reference)	1.00 (reference)	1.00 (reference)	1.00 (reference)	1.00 (reference)
Obesity	2.11 (1.88, 2.37)	1.32 (1.24, 1.40)	1.33 (1.25, 1.41)	2.02 (1.82, 2.24)	1.51 (1.42, 1.60)	1.51 (1.42, 1.60)	2.02 (1.88, 2.18)	1.42 (1.37, 1.48)	1.42 (1.36, 1.48)

BMI: body mass index; WC: waist circle; DBP: diastolic blood pressure; SBP: systolic blood pressure; OR: odds ratios; CI: confidence interval. (1) In model one: ^a^unadjusted, age-adjusted by design. (2) In model two: ^b^adjusted for age, education, marital status, living place, and BMI; ^d^adjusted for age, education, marital status, living place, and WC; ^f^adjusted for age, education, marital status, living place, and famine exposure. (3) In model three: ^c^adjusted for age, education, marital status, living place, smoking status, drinking status, eating habit, social activities, the experience of traumatic events, taking physical activity or exercise, and BMI; ^e^adjusted for age, education, marital status, living place, smoking status, drinking status, eating habit, social activities, the experience of traumatic events, taking physical activity or exercise, and WC; ^g^adjusted for age, education, marital status, living place, smoking status, drinking status, eating habit, social activities, the experience of traumatic events, taking physical activity or exercise, and famine exposure.

**Table 4:** Combined associations of obesity parameters and famine exposure with the prevalence of hypertension in male.

Famine exposure	OR and 95% CI for hypertension											
	Model one^a^				Model two^b^				Model three^c^			
	BMI levels				BMI levels				BMI levels			
	Underweight and normal	Overweight	Obesity	*P* for trend	Underweight and normal	Overweight	Obesity	*P* for trend	Underweight and normal	Overweight	Obesity	*P* for trend
No-exposed	1.0 0(reference)	2.08 (1.41, 3.06)	5.53 (3.44, 8.89)	<0.001	1.00 (reference)	2.07 (1.40, 3.05)	5.52 (3.43, 8.89)	<0.001	1.00 (reference)	2.11 (1.43, 3.11)	5.65 (3.50, 9.11)	<0.001
Fetal-exposed	1.43 (1.00, 2.05)	3.11 (2.10, 4.62)	5.49 (3.18, 9.48)	<0.001	1.42 (0.99, 2.03)	3.14 (2.12, 4.66)	5.41 (3.13, 9.36)	<0.001	1.40 (0.97, 2.00)	3.18 (2.14, 4.73)	5.38 (3.10, 9.31)	<0.001
Childhood-exposed	1.93 (1.45, 2.58)	3.65 (2.69, 4.97)	4.24 (2.88, 6.24)	<0.001	1.90 (1.43, 2.54)	3.61 (2.65, 4.92)	4.14 (2.81, 6.10)	<0.001	1.88 (1.41, 2.51)	3.70 (2.71, 5.04)	4.28 (2.90, 6.32)	<0.001
Adolescence/adult-exposed	3.12 (2.35, 4.13)	5.08 (3.70, 6.98)	7.38 (4.81, 11.32)	<0.001	2.94 (2.21, 3.90)	4.84 (3.52, 6.66)	6.87 (4.47, 10.57)	<0.001	3.00 (2.25, 3.99)	5.07 (3.67, 6.99)	7.30 (4.74, 11.25)	<0.001
*P* for trend	<0.001	<0.001	0.201		<0.001	<0.001	0.637		<0.001	<0.001	0.812	
*P* interaction		<0.001				<0.001				<0.001		
	WC levels				WC levels				WC levels			
	Normal	Central obesity			Normal	Central obesity			Normal	Central obesity		
No-exposed	1.0 0(reference)	3.78 (2.67, 5.36)			1.00 (reference)	3.77 (2.66, 5.35)			1.00 (reference)	3.81 (2.69, 5.41)		
Fetal-exposed	1.69 (1.2, 2.37)	4.00 (2.76, 5.81)			1.68 (1.20, 2.36)	4.00 (2.75, 5.81)			3.99 (2.75, 5.80)	2.01 (1.52, 2.66)		
Childhood-exposed	2.06 (1.56, 2.71)	4.57 (3.40, 6.13)			2.03 (1.54, 2.68)	4.47 (3.33, 6.00)			3.18 (2.41, 4.19)	5.97 (4.41, 8.08)		
Adolescence/adult-exposed	3.30 (2.51, 4.34)	6.13 (4.54, 8.26)			3.13 (2.38, 4.13)	5.75 (4.26, 7.77)			4.83 (3.63, 6.43)	6.68 (4.92, 9.07)		
*P* for trend	<0.001	<0.001			<0.001	<0.001			<0.001	<0.001		
*P* interaction	<0.001				<0.001				<0.001			

BMI: body mass index; WC: waist circle; DBP: diastolic blood pressure; SBP: systolic blood pressure; OR: odds ratios; CI: confidence interval. ^a^Unadjusted; age-adjusted by design. ^b^Adjusted for age, education, marital status, and living place. ^c^Adjusted for age, education, marital status, living place, smoking status, drinking status, eating habit, social activities, the experience of traumatic events, and taking physical activity or exercise.

**Table 5:** Combined associations of obesity parameters and famine exposure with the prevalence of hypertension in female.

Famine exposure	OR and 95% CI for hypertension											
	Model one^a^				Model two^b^				Model three^c^			
	BMI levels				BMI levels				BMI levels			
	Underweight and normal	Overweight	Obesity	*P* for trend	Underweight and normal	Overweight	Obesity	*P* for trend	Underweight and normal	Overweight	Obesity	*P* for trend
No-exposed	1.00 (reference)	2.03 (1.44, 2.87)	3.68 (2.48, 5.46)	<0.001	1.00 (reference)	2.03 (1.44, 2.87)	3.69 (2.48, 5.48)	<0.001	1.00 (reference)	2.03 (1.44, 2.87)	3.69 (2.48, 5.48)	<0.001
Fetal-exposed	1.29 (0.89, 1.88)	2.55 (1.79, 3.61)	4.08 (2.65, 6.28)	<0.001	1.28 (0.88, 1.86)	2.52 (1.78, 3.58)	4.05 (2.63, 6.23)	<0.001	1.29 (0.89, 1.87)	2.55 (1.80, 3.63)	4.10 (2.66, 6.31)	<0.001
Childhood-exposed	1.98 (1.49, 2.63)	3.45 (2.58, 4.62)	6.24 (4.52, 8.61)	<0.001	1.84 (1.39, 2.45)	3.21 (2.40, 4.31)	5.85 (4.23, 8.08)	<0.001	1.87 (1.40, 2.48)	3.24 (2.41, 4.34)	5.85 (4.23, 8.09)	<0.001
Adolescence/adult-exposed	5.73 (4.35, 7.56)	7.51 (5.56, 10.15)	10.38 (7.26, 14.84)	<0.001	4.82 (3.63, 6.41)	6.63 (4.89, 8.99)	8.88 (6.18, 12.75)	<0.001	4.83 (3.63, 6.43)	6.68 (4.92, 9.07)	8.89 (6.19, 12.78)	<0.001
*P* for trend	<0.001	<0.001	<0.001		<0.001	<0.001	<0.001		<0.001	<0.001	<0.001	
*P* interaction		<0.001				<0.001				<0.001		
	WC levels				WC levels				WC levels			
	Normal	Central obesity			Normal	Central obesity			Normal	Central obesity		
No-exposed	1.00 (reference)	2.39 (1.77, 3.24)			1.00 (reference)	2.41 (1.78, 3.26)			1.00 (reference)	2.39 (1.76, 3.24)		
Fetal-exposed	1.16 (0.82, 1.65)	2.89 (2.12, 3.93)			1.15 (0.81, 1.64)	2.87 (2.11,3.91)			1.16 (0.81, 1.65)	2.89 (2.12, 3.94)		
Childhood-exposed	1.75 (1.34, 2.29)	3.75 (2.90, 4.84)			1.65 (1.26, 2.16)	3.51 (2.71, 4.55)			1.66 (1.27, 2.18)	3.52 (2.71, 4.56)		
Adolescence/adult-exposed	4.68 (3.59, 6.1)	7.59 (5.86, 9.84)			4.03 (3.06, 5.29)	6.58 (5.05, 8.58)			4.03 (3.07, 5.31)	6.59 (5.05, 8.59)		
*P* for trend	<0.001	<0.001			<0.001	<0.001			<0.001	<0.001		
*P* interaction	<0.001				<0.001				<0.001			

BMI: body mass index; WC: waist circle; DBP: diastolic blood pressure; SBP: systolic blood pressure; OR: odds ratios; CI: confidence interval. ^a^Unadjusted; age-adjusted by design. ^b^Adjusted for age, education, marital status, and living place. ^c^Adjusted for age, education, marital status, living place, smoking status, drinking status, eating habit, social activities, the experience of traumatic events, and taking physical activity or exercise.

**Table 6:** Combined associations of obesity parameters and famine exposure with the prevalence of hypertension in total population.

Famine exposure	OR and 95% CI for hypertension											
	Model one^a^				Model two^b^				Model three^c^			
	BMI levels				BMI levels				BMI levels			
	Underweight and normal	Overweight	Obesity	*P* for trend	Underweight and normal	Overweight	Obesity	*P* for trend	Underweight and normal	Overweight	Obesity	*P* for trend
No-exposed	1.00 (reference)	2.02 (1.57, 2.62)	4.18 (3.10, 5.65)	<0.001	1.00 (reference)	2.03 (1.57, 2.62)	4.19 (3.1, 5.67)	<0.001	1.00 (reference)	2.06 (1.59, 2.67)	4.25 (3.14, 5.75)	<0.001
Fetal-exposed	1.38 (1.07, 1.78)	2.72 (2.09, 3.53)	4.42 (3.16, 6.17)	<0.001	1.36 (1.05, 1.77)	2.73 (2.1, 3.54)	4.38 (3.13, 6.13)	<0.001	1.36 (1.05, 1.76)	2.76 (2.12, 3.58)	4.44 (3.18, 6.21)	<0.001
Childhood-exposed	1.98 (1.62, 2.42)	3.52 (2.85, 4.35)	5.37 (4.21, 6.8 5)	<0.001	1.89 (1.55, 2.32)	3.37 (2.73, 4.17)	5.14 (4.02, 6.56)	<0.001	1.89 (1.54, 2.32)	3.43 (2.78, 4.24)	5.24 (4.10, 6.70)	<0.001
Adolescence/adult-exposed	4.16 (3.42, 5.07)	6.28 (5.05, 7.81)	9.04 (6.89, 11.86)	<0.001	3.67 (3.01, 4.49)	5.69 (4.57, 7.1)	7.94 (6.03, 10.44)	<0.001	3.69 (3.02, 4.52)	5.81 (4.66, 7.24)	8.13 (6.18, 10.71)	<0.001
*P* for trend	<0.001	<0.001	<0.001		<0.001	<0.001	<0.001		<0.001	<0.001	<0.001	
*P* interaction		<0.001				<0.001				<0.001		
	WC levels				WC levels				WC levels			
	Normal	Central obesity			Normal	Central obesity			Normal	Central obesity		
No-exposed	1.00 (reference)	2.84 (2.26, 3.57)			1.00 (reference)	2.88 (2.29, 3.62)			1.00 (reference)	2.90 (2.30, 3.64)		
Fetal-exposed	1.42 (1.12, 1.82)	3.23 (2.55, 4.09)			1.41 (1.11, 1.80)	3.26 (2.57, 4.13)			1.41 (1.10, 1.79)	3.27 (2.58, 4.14)		
Childhood-exposed	1.93 (1.59, 2.33)	4.01 (3.31, 4.86)			1.84 (1.52, 2.23)	3.87 (3.19, 4.7)			1.84 (1.52, 2.23)	3.91 (3.22, 4.74)		
Adolescence/adult-exposed	3.77 (3.12, 4.56)	7.05 (5.80, 8.56)			3.37 (2.78, 4.08)	6.29 (5.16, 7.66)			3.38 (2.78, 4.09)	6.36 (5.22, 7.75)		
*P* for trend	<0.001	<0.001			<0.001	<0.001			<0.001	<0.001		
*P* interaction	<0.001				<0.001				<0.001			

BMI: body mass index; WC: waist circle; DBP: diastolic blood pressure; SBP: systolic blood pressure; OR: odds ratios; CI: confidence interval. ^a^Unadjusted; age-adjusted by design. ^b^Adjusted for age, sex, education, marital status, and living place. ^c^Adjusted for age, sex, education, marital status, living place, smoking status, drinking status, eating habit, social activities, experience of traumatic events, and taking physical activity or exercise.

## Data Availability

All data are openly published as microdata at http://charls.pku.edu.cn/index/zh-cn.html with no direct contact with all participants.

## Abbreviations

WHO: World Health Organization
CHARLS: China Health and Retirement Longitudinal Study
BMI: Body mass index
WC: Waist circle
BP: Blood pressure
DBP: Diastolic blood pressure
SBP: Systolic blood pressure
M: Mean
B: Unstandardized
CDC: Centers for Disease Control and Prevention
NSFC: The National Natural Science Foundation of China
NIA: National Institute on Aging
WB: World Bank
UA: Urinalysis.

## References

[1] de Kouchkovsky I., Mayfield J., Kohlwes J. (2019). Hypertension in young adults and subsequent cardiovascular disease. *JAMA*.

[2] Gutierrez J., Alloubani A., Mari M., Alzaatreh M. (2018). Cardiovascular disease risk factors: hypertension, diabetes mellitus and obesity among Tabuk citizens in Saudi Arabia. *Open Cardiovascular Medicine Journal*.

[3] James J. E. (2017). Hypertension control and cardiovascular disease. *Lancet*.

[4] Abdulsalam S., Olugbenga-Bello A., Olarewaju O., Abdus-Salam I. (2014). Sociodemographic correlates of modifiable risk factors for hypertension in a rural local government area of Oyo state south west Nigeria. *International Journal of Hypertension*.

[5] Ke L., Ho J., Feng J. (2014). Modifiable risk factors including sunlight exposure and fish consumption are associated with risk of hypertension in a large representative population from Macau. *The Journal of Steroid Biochemistry and Molecular Biology*.

[6] Ibekwe R. (2015). Modifiable risk factors of hypertension and socio-demographic profile in Oghara, delta state; prevalence and correlates. *Annals of Medical and Health Sciences Research*.

[7] Pilakkadavath Z., Shaffi M. (2016). Modifiable risk factors of hypertension: a hospital-based case-control study from Kerala, India. *Journal of Family Medicine and Primary Care*.

[8] Mamudu H. M., Paul T. K., Wang L. (2017). Association between multiple modifiable risk factors of cardiovascular disease and hypertension among asymptomatic patients in central Appalachia. *Southern Medical Journal*.

[9] Gluckman P. D., Hanson M. A., Cooper C., Thornburg K. L. (2008). Effect of in utero and early-life conditions on adult health and disease. *The New England Journal of Medicine*.

[10] Alexander B. T. (2006). Fetal programming of hypertension. *American Journal of Physiology-Regulatory, Integrative and Comparative Physiology*.

[11] Li Y., Jaddoe V. W., Qi L. (2011). Exposure to the Chinese famine in early life and the risk of hypertension in adulthood. *Journal of Hypertension*.

[12] van Abeelen A. F. M., de Rooij S. R., Osmond C. (2011). The sex-specific effects of famine on the association between placental size and later hypertension. *Placenta*.

[13] Carroll D., Ginty A. T., Painter R. C., Roseboom T. J., Phillips A. C., de Rooij S. R. (2012). Systolic blood pressure reactions to acute stress are associated with future hypertension status in the Dutch Famine Birth Cohort Study. *International Journal of Psychophysiology: official journal of the International Organization of Psychophysiology*.

[14] Wang P. X., Wang J. J., Lei Y. X., Xiao L., Luo Z. C. (2012). Impact of fetal and infant exposure to the Chinese Great Famine on the risk of hypertension in adulthood. *PLoS One*.

[15] Chen H., Nembhard W. N., Stockwell H. G. (2014). Sex-specific effects of fetal exposure to the 1959-1961 Chinese famine on risk of adult hypertension. *Maternal and Child Health Journal*.

[16] Wang Z., Li C., Yang Z., Zou Z., Ma J. (2016). Infant exposure to Chinese famine increased the risk of hypertension in adulthood: results from the China Health and Retirement Longitudinal Study. *BMC Public Health*.

[17] Liu L., Xu X., Zeng H. (2017). Increase in the prevalence of hypertension among adults exposed to the Great Chinese Famine during early life. *Environmental Health and Preventive Medicine*.

[18] Wu L., Feng X., He A., Ding Y., Zhou X., Xu Z. (2017). Prenatal exposure to the Great Chinese Famine and mid-age hypertension. *PLoS One*.

[19] Yu C., Wang J., Li Y. (2017). Exposure to the Chinese famine in early life and hypertension prevalence risk in adults. *PLoS One*.

[20] Liu L., Xu X., Zeng H. (2018). Correction to: increase in the prevalence of hypertension among adults exposed to the great Chinese famine during early life. *Environmental Health and Preventive Medicine*.

[21] Shi Z., Nicholls S. J., Taylor A. W., Magliano D. J., Appleton S., Zimmet P. (2018). Early life exposure to Chinese famine modifies the association between hypertension and cardiovascular disease. *Journal of Hypertension*.

[22] Xin X., Yao J., Yang F., Zhang D. (2018). Famine exposure during early life and risk of hypertension in adulthood: a meta-analysis. *Critical Reviews in Food Science and Nutrition*.

[23] Zhao R., Duan X., Wu Y., Zhang Q., Chen Y. (2019). Association of exposure to Chinese famine in early life with the incidence of hypertension in adulthood: a 22-year cohort study. *Nutrition, Metabolism, and Cardiovascular Diseases: NMCD*.

[24] Chen J. P., Peng B., Tang L. (2016). Fetal and infant exposure to the Chinese famine increases the risk of fatty liver disease in Chongqing, China. *Journal of Gastroenterology and Hepatology*.

[25] Zhou J., Sheng J., Fan Y. (2019). The effect of Chinese famine exposure in early life on dietary patterns and chronic diseases of adults. *Public Health Nutrition*.

[26] Liu L., Pang Z. C., Sun J. P. (2017). Exposure to famine in early life and the risk of obesity in adulthood in Qingdao: evidence from the 1959-1961 Chinese famine. *Nutrition, Metabolism, and Cardiovascular Diseases: NMCD*.

[27] Chang X., Song P., Wang M., An L. (2018). The risks of overweight, obesity and abdominal obesity in middle age after exposure to famine in early life: evidence from the China’s 1959-1961 famine. *The Journal of Nutrition, Health & Aging*.

[28] Meng R., Lv J., Yu C. (2018). Prenatal famine exposure, adulthood obesity patterns and risk of type 2 diabetes. *International Journal of Epidemiology*.

[29] Zhou J., Zhang L., Xuan P. (2018). The relationship between famine exposure during early life and body mass index in adulthood: a systematic review and meta-analysis. *PLoS One*.

[30] Fang Z., Chen C., Wang H., Tang K. (2020). Association between fetal exposure to famine and anthropometric measures in adulthood: a regression discontinuity approach. *Obesity*.

[31] Song C., Wang M., Chen Z. (2020). Fetal exposure to Chinese famine increases obesity risk in adulthood. *International Journal of Environmental Research and Public Health*.

[32] Li C., Liu T., Sun W., Wu L., Zou Z. Y. (2015). Prevalence and risk factors of arthritis in a middle-aged and older Chinese population: the China health and retirement longitudinal study. *Rheumatology*.

[33] Zhang L., Liu K., Li H. (2016). Relationship between body mass index and depressive symptoms: the “fat and jolly” hypothesis for the middle-aged and elderly in China. *BMC Public Health*.

[34] Zhang L., Li J. L., Zhang L. L., Guo L. L., Li H., Li D. (2018). No association between C-reactive protein and depressive symptoms among the middle-aged and elderly in China Evidence from the China Health and Retirement Longitudinal Study. *Medicine*.

[35] Zhang L., Yang L., Wang C. (2021). Individual and combined association analysis of famine exposure and serum uric acid with hypertension in the mid-aged and older adult: a population-based cross-sectional study. *BMC Cardiovascular Disorders*.

[36] Zhang L., Li J. L., Zhang L. L. (2019). Relationship between adiposity parameters and cognition: the “fat and jolly” hypothesis in middle-aged and elderly people in China. *Medicine*.

[37] Zhang L., Li J. L., Zhang L. L., Guo L. L., Li H., Li D. (2020). Body mass index and serum uric acid level. *Medicine (Baltimore)*.

[38] Zhang L., Li J. L., Guo L. L., Li H., Li D., Xu G. (2020). The interaction between serum uric acid and triglycerides level on blood pressure in middle-aged and elderly individuals in China: result from a large national cohort study. *BMC Cardiovascular Disorders*.

[39] Zhou B. F. (2002). Effect of body mass index on all-cause mortality and incidence of cardiovascular diseases--report for meta-analysis of prospective studies open optimal cut-off points of body mass index in Chinese adults. *Biomedical and Environmental Sciences: BES*.

[40] Zhou H. C., Lai Y. X., Shan Z. Y. (2014). Effectiveness of different waist circumference cut-off values in predicting metabolic syndrome prevalence and risk factors in adults in China. *Biomedical and Environmental Sciences: BES*.

[41] Wang N., Wang X., Li Q. (2017). The famine exposure in early life and metabolic syndrome in adulthood. *Clinical Nutrition (Edinburgh, Scotland)*.

[42] Li Y., Zhao L., Yu D., Ding G. (2018). Exposure to the Chinese famine in early life and depression in adulthood. *Psychology, Health & Medicine*.

[43] Song S. (2009). Does famine have a long-term effect on cohort mortality? Evidence from the 1959-1961 great leap forward famine in China. *Journal of Biosocial Science*.

[44] de Rooij S. R., Painter R. C., Holleman F., Bossuyt P. M., Roseboom T. J. (2007). The metabolic syndrome in adults prenatally exposed to the Dutch famine. *The American Journal of Clinical Nutrition*.

[45] Stein A. D., Zybert P. A., van der Pal-de Bruin K., Lumey L. H. (2006). Exposure to famine during gestation, size at birth, and blood pressure at age 59 y: evidence from the Dutch famine. *European Journal of Epidemiology*.

[46] Stanner S. A., Bulmer K., Andrès C. (1997). Does malnutrition in utero determine diabetes and coronary heart disease in adulthood? Results from the Leningrad siege study, a cross sectional study. *BMJ*.

[47] Khanal P., Johnsen L., Axel A. M. (2016). Long-term impacts of foetal malnutrition followed by early postnatal obesity on fat distribution pattern and metabolic adaptability in adult sheep. *PLoS One*.

[48] Bol V., Desjardins F., Reusens B., Balligand J. L., Remacle C. (2010). Does early mismatched nutrition predispose to hypertension and atherosclerosis, in male mice?,. *PloS One*.

[49] Bai S. Y., Briggs D. I., Vickers M. H. (2012). Increased systolic blood pressure in rat offspring following a maternal low-protein diet is normalized by maternal dietary choline supplementation. *Journal of Developmental Origins of Health and Disease*.

[50] Kubaszek A., Markkanen A., Eriksson J. G. (2004). The association of the K121Q polymorphism of the plasma cell glycoprotein-1 gene with type 2 diabetes and hypertension depends on size at birth. *The Journal of Clinical Endocrinology and Metabolism*.

[51] Aagaard-Tillery K. M., Grove K., Bishop J. (2008). Developmental origins of disease and determinants of chromatin structure: maternal diet modifies the primate fetal epigenome. *Journal of Molecular Endocrinology*.

[52] Singhal A., Lucas A. (2004). Early origins of cardiovascular disease: is there a unifying hypothesis?. *Lancet*.

[53] Peng Y., Hai M., Li P., Chen Y. (2020). Association of exposure to Chinese famine in early life with the risk of metabolic syndrome in adulthood. *Annals of Nutrition & Metabolism*.

[54] Feng X. L., Liu J. H., Yan S. (2020). Prenatal exposure to the Chinese famine and the risk of metabolic syndrome in adulthood across consecutive generations. *Journal of Diabetes Research*.

[55] Ning F., Ren J., Song X. (2019). Famine exposure in early life and risk of metabolic syndrome in adulthood: comparisons of different metabolic syndrome definitions.

[56] Zheng X., Wang Y., Ren W. (2012). Risk of metabolic syndrome in adults exposed to the great Chinese famine during the fetal life and early childhood. *European Journal of Clinical Nutrition*.

[57] Li Y., Jaddoe V. W., Qi L. (2011). Exposure to the chinese famine in early life and the risk of metabolic syndrome in adulthood. *Diabetes Care*.

[58] Ma R. C. W., Zimmet P., Liu H. (2020). Association of famine exposure with the risk of type 2 diabetes: a meta-analysis. *Journal of Diabetes*.

[59] Lu J. (2020). Early life famine exposure, ideal cardiovascular health metrics, and risk of incident diabetes: findings from the 4C study. *The British Journal of Nutrition*.

[60] Ji L., Shi Z. (2020). Early life exposure to 1959-1961 Chinese famine exacerbates association between diabetes and cardiovascular disease. *Nature Reviews. Endocrinology*.

[61] Hu X., Wen J., Yu W. (2021). Associations of early-life exposure to famine with abdominal fat accumulation are independent of family history of diabetes and physical activity. *British Journal of Nutrition*.

[62] Li C., Tobi E. W., Heijmans B. T., Lumey L. H. (2019). The effect of the Chinese famine on type 2 diabetes mellitus epidemics. *Nature Reviews Endocrinology*.

[63] Li C., Lumey L. H. (2019). Interaction or mediation by adult obesity of the relation between fetal famine exposure and type 2 diabetes?. *Nature Reviews Endocrinology*.

[64] Wang Z., Zou Z., Yang Z. (2018). The association between fetal-stage exposure to the China famine and risk of diabetes mellitus in adulthood: results from the China health and retirement longitudinal study. *BMC Public Health*.

[65] Sun Y., Zhang L., Duan W., Meng X., Jia C. (2018). Association between famine exposure in early life and type 2 diabetes mellitus and hyperglycemia in adulthood: results from the China Health And Retirement Longitudinal Study(CHARLS). *Journal of Diabetes*.

[66] Li T., Zhang Y., Wang J. (2018). All-cause mortality risk associated with long-term exposure to ambient PM_2_ _∗__5_ in China: a cohort study. *The Lancet Public health*.

[67] Wang N., Cheng J., Han B. (2017). Exposure to severe famine in the prenatal or postnatal period and the development of diabetes in adulthood: an observational study. *Diabetologia*.

[68] Li J., Liu S., Li S. (2017). Prenatal exposure to famine and the development of hyperglycemia and type 2 diabetes in adulthood across consecutive generations: a population-based cohort study of families in Suihua, China. *The American Journal of Clinical Nutrition*.

[69] Wang J., Li Y., Han X. (2016). Exposure to the Chinese famine in childhood increases type 2 diabetes risk in adults. *The Journal of Nutrition*.

[70] Lumey L. H., Khalangot M. D., Vaiserman A. M. (2015). Association between type 2 diabetes and prenatal exposure to the Ukraine famine of 1932-33: a retrospective cohort study. *The Lancet. Diabetes & Endocrinology*.

[71] van Abeelen A. F., Elias S. G., Bossuyt P. M. (2012). Famine exposure in the young and the risk of type 2 diabetes in adulthood. *Diabetes*.

[72] Portrait F., Teeuwiszen E., Deeg D. (1982). Early life undernutrition and chronic diseases at older ages: the effects of the Dutch famine on cardiovascular diseases and diabetes. *Social Science & Medicine*.

[73] Li Y., He Y., Qi L. (2010). Exposure to the Chinese famine in early life and the risk of hyperglycemia and type 2 diabetes in adulthood. *Diabetes*.

[74] Arage G., Belachew T., Abera M., Abdulhay F., Abdulahi M., Hassen Abate K. (2020). Consequences of early life exposure to the 1983-1985 Ethiopian great famine on cognitive function in adults: a historical cohort study. *BMJ Open*.

[75] Rong H., Lai X., Mahmoudi E., Fang H. (2019). Early-life exposure to the Chinese famine and risk of cognitive decline. *Journal of Clinical Medicine*.

[76] Li C., Miles T., Shen L. (2018). Early-life exposure to severe famine and subsequent risk of depressive symptoms in late adulthood: the China Health and Retirement Longitudinal Study. *The British Journal of Psychiatry: the Journal of Mental Science*.

[77] He P., Liu L., Salas J. M. I. (2018). Prenatal malnutrition and adult cognitive impairment: a natural experiment from the 1959-1961 Chinese famine. *The British Journal of Nutrition*.

[78] Rong H., Xi Y., An Y. (2017). The correlation between early stages of life exposed to Chinese famine and cognitive decline in adulthood: nutrition of adulthood plays an important role in the link?. *Frontiers in Aging Neuroscience*.

[79] Wang C., An Y., Yu H. (2016). Association between exposure to the Chinese famine in different stages of early life and decline in cognitive functioning in adulthood. *Frontiers in Behavioral Neuroscience*.

[80] Li J., Na L., Ma H. (2015). Multigenerational effects of parental prenatal exposure to famine on adult offspring cognitive function. *Scientific Reports*.

[81] He S., Li J., Wang Z. (2020). Early-life exposure to famine and late-life depression: does leukocyte telomere length mediate the association?. *Journal of Affective Disorders*.

[82] Stein A. D., Pierik F. H., Verrips G. H., Susser E. S., Lumey L. H. (2009). Maternal exposure to the Dutch famine before conception and during Pregnancy. *Epidemiology*.

[83] Zhang L., Li J. L., Zhang L. L., Guo L. L., Li H., Li D. (2018). Association and interaction analysis of body mass index and triglycerides level with blood pressure in elderly individuals in China. *BioMed Research International*.

[84] Sun H., Ren X., Chen Z. (2016). Association between body mass index and mortality in a prospective cohort of Chinese adults. *Medicine (Baltimore)*.

[85] Hu J., Xu H., Zhu J. (2021). Association between body mass index and risk of cardiovascular disease-specific mortality among adults with hypertension in Shanghai, China. *Aging*.

[86] Kim N. H., Lee J., Kim T. J. (2015). Body mass index and mortality in the general population and in subjects with chronic disease in Korea: a nationwide cohort study (2002-2010). *PLoS One*.

[87] Li K., Yao C., Yang X. (2016). Body mass index and the risk of cardiovascular and all-cause mortality among patients with hypertension: a population-based prospective cohort study among adults in Beijing, China. *Journal of Epidemiology*.

[88] Nguyen Q. N., Pham S. T., Nguyen V. L. (2012). Time trends in blood pressure, body mass index and smoking in the Vietnamese population: a meta-analysis from multiple cross-sectional surveys. *PLoS One*.

[89] Power B. D., Alfonso H., Flicker L., Hankey G. J., Yeap B. B., Almeida O. P. (2011). Body adiposity in later life and the incidence of dementia: the health in men study. *PLoS One*.

[90] Ferra A., del Mar Bibiloni M., Zapata M. E., Pich J., Pons A., Tur J. A. (2012). Body mass index, life-style, and healthy status in free living elderly people in Menorca Island. *The Journal of Nutrition, Health & Aging*.

[91] Oxlund C. S., Pareek M., Rasmussen B. S. B. (2019). Body mass index, intensive blood pressure management, and cardiovascular events in the SPRINT trial. *The American Journal of Medicine*.

[92] Cox B. D., Whichelow M. J., Prevost A. T. (1998). The development of cardiovascular disease in relation to anthropometric indices and hypertension in British adults. *International Journal of Obesity and Related Metabolic Disorders: Journal of the International Association for the Study of Obesity*.

[93] Atella V., Kopinska J., Medea G. (2015). Excess body weight increases the burden of age-associated chronic diseases and their associated health care expenditures. *Aging*.

[94] Ramirez S. P., McClellan W., Port F. K., Hsu S. I. (2002). Risk factors for proteinuria in a large, multiracial, southeast Asian population. *Journal of the American Society of Nephrology: JASN*.

[95] van Uffelen J. G., Berecki-Gisolf J., Brown W. J., Dobson A. J. (2010). What is a healthy body mass index for women in their seventies? Results from the Australian longitudinal study on women’s Health. *The Journals of Gerontology Series A: Biological Sciences and Medical Sciences*.

[96] Yang W., Li J. P., Zhang Y. (2016). Association between Body Mass Index and All-Cause Mortality in Hypertensive Adults: Results from the China Stroke Primary Prevention Trial (CSPPT). *Nutrients*.

[97] Burgos L. M., Gil Ramírez A., Seoane L. (2021). Is the obesity paradox in cardiac surgery really a myth? Effect of body mass index on early and late clinical outcomes. *Journal of Cardiothoracic and Vascular Anesthesia*.

[98] Dwivedi A. K., Dubey P., Cistola D. P., Reddy S. Y. (2020). Association between obesity and cardiovascular outcomes: updated evidence from meta-analysis studies. *Current Cardiology Reports*.

